# Gastrointestinal Tract Disease Classification from Wireless Endoscopy Images Using Pretrained Deep Learning Model

**DOI:** 10.1155/2021/5940433

**Published:** 2021-09-11

**Authors:** J. Yogapriya, Venkatesan Chandran, M. G. Sumithra, P. Anitha, P. Jenopaul, C. Suresh Gnana Dhas

**Affiliations:** ^1^Department of Computer Science and Engineering, Kongunadu College of Engineering and Technology, Trichy, 621215 Tamil Nadu, India; ^2^Department of Electronics and Communication Engineering, Dr.N.G.P Institute of Technology, Coimbatore, 641048 Tamilnadu, India; ^3^Department of Biomedical Engineering, Dr.N.G.P Institute of Technology, Coimbatore, 641048 Tamilnadu, India; ^4^Department of EEE, Adi Shankra Institute of Engineering and Technology, Kalady, Ernakulam, Kerala 683574, India; ^5^Department of Computer Science, Ambo University, Ambo University, Ambo, Post Box No.: 19, Ethiopia

## Abstract

Wireless capsule endoscopy is a noninvasive wireless imaging technology that becomes increasingly popular in recent years. One of the major drawbacks of this technology is that it generates a large number of photos that must be analyzed by medical personnel, which takes time. Various research groups have proposed different image processing and machine learning techniques to classify gastrointestinal tract diseases in recent years. Traditional image processing algorithms and a data augmentation technique are combined with an adjusted pretrained deep convolutional neural network to classify diseases in the gastrointestinal tract from wireless endoscopy images in this research. We take advantage of pretrained models VGG16, ResNet-18, and GoogLeNet, a convolutional neural network (CNN) model with adjusted fully connected and output layers. The proposed models are validated with a dataset consisting of 6702 images of 8 classes. The VGG16 model achieved the highest results with 96.33% accuracy, 96.37% recall, 96.5% precision, and 96.5% F1-measure. Compared to other state-of-the-art models, the VGG16 model has the highest Matthews Correlation Coefficient value of 0.95 and Cohen's kappa score of 0.96.

## 1. Introduction

Esophageal, stomach, and colorectal cancers account for 2.8 million new cases and 1.8 million deaths worldwide per year. Out of these ulcers, bleeding and polyps are all examples of gastrointestinal infections [1]. Since the beginning of 2019, an estimated 27,510 cases have been diagnosed in the United States, with 62.63% males and 37.37% females, and estimated deaths of 40.49%, with 61% males and 39% females [2]. Due to its complex nature, gastroscopy instruments are not suitable for identifying and examining gastrointestinal infections such as bleeding, polyps, and ulcers. In the year 2000, wireless capsule endoscopy (WCE) was developed to solve the problem with gastroscopy instruments [3]. Conferring to the yearly report in 2018, roughly 1 million patients were successfully treated with the assistance of WCE [4]. To detect disease, the doctor employs the WCE procedure to inspect the interior of the gastrointestinal tract (GIT). The doctor uses the WCE method to inspect the interior of the gastrointestinal tract in order to discover disease (GIT) [5, 6]. The capsule autonomously glides across the GI tract, giving real-time video to the clinician. After the process of transmitting the videos, the capsule is discharged through the anus. The video frames received are examined by the physician to decide about the diseases [7]. The major diseases diagnosed using the WCE are ulcers, bleeding, malignancy, and polyps in the digestive system. The anatomical landmarks, pathological findings, and poly removal play a vital role in diagnosing the diseases in the digestive system using WCE captured images. It is a more convenient method to diagnose by providing a wide range of visuals [8]. It reduces the patient's discomfort and complications during the treatment in conventional endoscopy methods like computer tomography enteroclysis and enteroscopy. The accuracy of diagnosing tumours and gastrointestinal bleeding, especially in the small intestine, has improved. The overall process is very time-consuming to analyze all the frames extracted from each patient [9]. Furthermore, even the most experienced physicians confront difficulties that necessitate a large amount of time to analyze all of the data because the contaminated zone in one frame will not emerge in the next. Even though the majority of the frames contain useless material, the physician must go through the entire video in order. Owing to inexperience or negligence, it may often result in a misdiagnosis [10].

Segmentation, classification, detection, and localization are techniques used to solve this problem by researchers. Feature extraction and visualization are an important step that determines the overall accuracy of the computer-aided diagnosis method. The different features are extracted based upon the texture analysis, color-based, points, and edges in the images [11]. The features extracted are insufficient to determine the model's overall accuracy. As a result, feature selection is a time-consuming process that is crucial in determining the model's output. The advancements in the field of deep learning, especially CNN, can solve the problem [12]. The advancement of CNN has been promising in the last decades, with automated detection of diseases in various organs of the human body, such as the brain [13], cervical cancer [14], eye diseases [15], and skin cancer [16]. Unlike conventional learning algorithms such as machine learning, the CNN model has the advantage of extracting features hierarchically from low to a high level. The remainder of the manuscript is organized as follows: Section 2 explains the related work in the field of GIT diagnosis; Section 3 discusses the dataset consider for this study; Section 4 describes the pretrained architecture to diagnose eight different diseases from WCE images; Section 5 contains the derived findings from the proposed method; Section 6 concludes the work.

## 2. Related Work

The automated prediction of anatomical landmarks, pathological observations, and polyp groups from images obtained using wireless capsule endoscopy is the subject of this research. The experimental groups from the pictures make it simple for medical experts to make an accurate diagnosis and prescribe a treatment plan. Significant research in this area has led to the automatic detection of infection from a large number of images, saving time and effort for medical experts while simultaneously boosting diagnosis accuracy. Automatically detecting infected image from WCE images has lately been a popular research topic, with a slew of papers published in the field. Traditional machine learning algorithms and deep learning algorithms are used in these studies. Improving the classification of disease areas with a high degree of precision in automatic detection is a great challenge. Advanced deep learning techniques are important in WCE to boost its analytical vintage. The AlexNet model is proposed to classify the upper gastrointestinal organs from the images captured under different conditions. The model achieves an accuracy of 96.5% in upper gastrointestinal anatomical classification [17]. The author proposed the technique to reduce the review time of endoscopy screening based on the analysis of factorization. The sliding window mechanism with single value decomposition is used. The technique achieves an overall precision of 92% [18]. The author proposed a system for automatically detecting irregular WCE images by extracting fractal features using the differential box-counting method. The output is tested on two datasets, both of which contain WCE frames, and achieves binary classification accuracy of 85% and 99% for dataset I and dataset II, respectively [19]. The author uses the pretrained models Inception-v4, Inception ResNet-v2, and NASNet to classify the anatomical landmarks from the WCE images, which obtained 98.45%, 98.48%, and 97.35%. Out of this, the Inception-v4 models achieves a precision of 93.8% [20]. To extract the features from the data, the authors used AlexNet and GoogLeNet. This approach is aimed at addressing the issues of low contrast and abnormal lesions in endoscopy [21]. The author proposed a computer-aided diagnostics tool for classifying ulcerative colitis and achieves the area under the curve of 0.86 for mayo 0 and 0.98 for mayo 0-1 [22]. The author proposed the convolutional neural network with four layers to classify a different class of ulcers from the WCE video frames. The test results are improved by tweaking the model's hyperparameters and achieving an accuracy of 96.8% [23]. The authors have introduced the new virtual reality capsule to simulate and identify the normal and abnormal regions. This environment is generated new 3D images for gastrointestinal diseases [24]. Local spatial features are retrieved from pixels of interest in a WCE image using a linear separation approach in this paper. The proposed probability density function model fitting-based approach not only reduces computing complexity, but it also results in a more consistent representation of a class. The proposed scheme performs admirably in terms of precision, with a score of 96.77% [25]. In [26], the author proposed a Gabor capsule network for classifying complex images like the Kvasir dataset. The model achieves an overall accuracy of 91.50%. The wavelet transform with a CNN is proposed to classify gastrointestinal tract diseases and achieves an overall average performance of 93.65% in classifying the eight classes [27].

From the literature, the CNN model can provide better results if the number of the dataset is high. But there are several obstacles in each step that will reduce the model's performance. The low contrast video frames in the dataset make segmenting the regions difficult. The extraction and selection of important traits are another difficult step in identifying disorders including ulcers, bleeding, and polyps. The workflow of the proposed method for disease classification using wireless endoscopy is shown in Figure 1. The significant contributions of this study are as follows.

1. A computer-assisted diagnostic system is being proposed to classify GIT diseases into many categories, including anatomical landmarks, pathological observations, and polyp removal
2. The pretrained model is used to overcome small datasets and overfitting problem, which reduces the model accuracy [28]
3. The VGG16, ResNet-18, and GoogLeNet pretrained CNN architecture classify gastrointestinal tract diseases from the endoscopic images by slightly modifying the architecture
4. The visual features of GIT disease ways of obtaining classification decisions are visualized using the occlusion sensitivity map
5. We also compared the modified pretrained architecture with other models, which used handcrafted features and in-depth features to detect the GIT diseases in accuracy, recall, precision, F1-measure, region of characteristics (ROC) curve, and Cohen's kappa score

## 3. Dataset Description

The dataset used in these studies is a GIT images taken with endoscopic equipment at Norway's VV health trust. The training data is obtained from a large gastroenterology department at one of the hospitals in this trust. The further medical experts meticulously annotated the dataset and named it Kvasir-V2. This dataset was made available in the fall of 2017 as part of the Mediaeval Medical Multimedia Challenge, a benchmarking project that assigns tasks to the research group [29]. Anatomical landmarks, pathological observations, and polyp removal are among the eight groups that make up the dataset with 1000 images each. The images in the dataset range in resolution from 720 × 576 to 1920 × 1072 pixels. The different diseases with corresponding class label encoding are provided in Table 1.

An anatomical landmark is a characteristic of the GIT that can be seen through an endoscope. It is necessary for navigation and as a reference point for describing the location of a given discovery. It is also possible that the landmarks are specific areas for pathology, such as ulcers or inflammation. Class 0 and class 1 are the two classes of poly removal. Class 3, class 4, and class 5 are the most important anatomical landmarks. The essential pathological findings are class 2, class 6, and class 7. The sample image from the dataset is shown in Figure 2, and the distribution of the dataset is represented in Figure 3.

## 4. Proposed Deep Learning Framework

To solve the issue of small data sizes, transfer learning was used to fine-tune three major pretrained deep neural networks called VGG16, ResNet-18, and GoogLeNet on the training images of the augmented Kvasir version 2 dataset.

### 4.1. Transfer Learning

In the world of medical imaging, classifying multiple diseases using the same deep learning architecture is a difficult task. Transfer learning is a technique for repurposing a model trained on one task to a comparable task that requires some adaptation. When there are not enough training samples to train a model from start, transfer learning is particularly beneficial for applications like medical picture classification for rare or developing diseases. This is particularly true for deep neural network models, which must be trained with a huge number of parameters. Transfer learning enables model parameters to start with good initial values that only need minimal tweaks to be better curated for the new problem. Transfer learning can be done in two ways; one approach is training the model from the top layers, and another approach is freezing the top layers of the model and fine-tunes it on the new dataset. The eight different types of diseases are considered in the proposed model, so the first approach is used where the model is trained from the top layers. VGG16, GoogLeNet, and ResNet-18 are the pretrained model used for classifying the different gastrointestinal tract diseases using endoscopic images. The above pretrained models are used as baseline models, and the model performance is increased by using various performance improvement techniques.

### 4.2. Gastrointestinal Tract Disease Classification Using VGG16

The VGG16 model comprises 16 layers which consist of 13 convolution layers and three dense layers. This model is initially introduced in 2014 for the ImageNet competition. The VGG16 is one of the best models for image classification.  Figure 4 depicts the architecture of the VGG16 model.

Instead of having many parameters, the model focuses on having a 3 × 3 convolution layer with stride one and padding that is always the same. The max-pooling layer uses a 2 × 2 filter with a stride of two. The model is completed by two dense layers, followed by the softmax layer. There are approximately 138 million parameters in the model [30]. The dense layers 1 and 2 consist of 4096 nodes. The dense layer 1 consists of a maximum number of parameters of 100 million approximately. The number of the parameter in that particular layer is reduced without degrading the performance of the model.

### 4.3. Gastrointestinal Tract Disease Classification Using ResNet-18

Another pretrained model for classifying gastrointestinal tract disease from endoscopic images is the ResNet-18 model.  Figure 5 depicts the architecture of the ResNet-18 platform. This model is based on a convolutional neural network, one of the most common architectures for efficient training. It allows for a smooth gradient flow. The identity shortcut link in the ResNet-18 model skips one or more layers. This will allow the network to have a narrow connection to the network's first layers, rendering gradient upgrades much easier for those layers [31]. The ResNet model comprises 17 convolution layers and one fully connected layer.

### 4.4. Gastrointestinal Tract Disease Classification Using GoogLeNet

In many transfer learning tasks, the GoogLeNet model is a deep CNN model that obtained good classification accuracy while improving compute efficiency. With a top-5 error rate of 6.67%, the GoogLeNet, commonly known as the Inception model, won the ImageNet competition in 2015. The inception module is shown in Figure 6, and the GoogLeNet architecture is shown in Figure 7. It has 22 layers, including 2 convolution layers, 4 max-pooling layers, and 9 linearly stacked inception modules. The average pooling is introduced at the end of the previous inception module. To execute the dimension reduction, the 1 × 1 filter is employed before the more expensive 3 × 3 and 5 × 5 operations. When compared to the AlexNet model, the GoogLeNet model has twice the amount of parameters.

### 4.5. Data Augmentation

The CNN models are proven to be suitable for many computer vision tasks; however, they required a considerable amount of training data to avoid overfitting. Overfitting occurs when a deep learning model learns a high-variance function that precisely models the training data but has a narrow range of generalizability. But in many cases, especially for medical image datasets obtained, a large amount of data is a tedious task. Different data augmentation techniques are used to increase the size and consistency of the data to solve the issue of overfitting. These techniques produce dummy data that has been subjected to different rotations, width changes, height shifts, zooming, and horizontal flip but is not the same as the original data. The rotation range is fixed as 45°, shifting width and height range is 0.2, zooming range of 0.2, and horizontal flip. The augmented dataset from the original Kvasir version 2 dataset is shown in Figure 8.

## 5. Results and Discussion

In this work, the Kvasir version 2 dataset is used for the classification of GIT diseases. The entire dataset is divided into an 80% training and 20% validation set. NVIDIA Digits uses the Caffe deep learning system to build the pretrained CNN models. The CNN pretrained model is trained and tested with a system configuration Intel i9 processor with 32 GB NVIDIA Quadro RTX6000 GPU. The pretrained models are written with the Caffe deep learning framework in the NVIDIA Digits platform. Images with resolutions ranging from 720 × 576 to 1920 × 1072 pixels were transformed to 256 × 256 pixels in the collected dataset. The augmented dataset is consisting of 33536 images which contained 4192 images in individual classes. Then, the augmented datasets are divided into 80% training and 20% validation set. There are 26832 images in the training and 6407 images in the validation. The pretrained models are trained from scratch with the hyperparameters of 30 epoch, batch size of 8, Adam optimizers, and learning rate of 1-*e*05 with step size 33% via trial and error method by considering the computing facility. The Adam optimizers are used due to their reduced complexity during the model training [32]. The softmax classification layer and categorical cross-entropy are used in the output of the pretrained model, and it is given in equations (1) and (2).

(1) $$\begin{array}{c} \sigma {\left(\bar{Z}\right)}_{i}=\frac{e^{z_{i}}}{\sum_{j=1}^{K}e^{z_{j}}}, \end{array}$$

where *σ* denotes the softmax,$\;\bar{Z}$ denotes the input vector, *e*^*z*_*i*_^ denotes the standard exponential of the input vector, *K* denotes the number of classes, and *e*^*z*_*j*_^ denotes the standard exponential of the output vector.

(2) $$\begin{array}{c} \text{Categorical Cross Entropy}=-\overset{\begin{array}{c} \text{Output}\\ \text{Size} \end{array}}{\underset{i=1}{\sum }}y_{i}.\log{\hat{y}}_{i}, \end{array}$$

where *y*_*i*_ denotes target value and $\hat{y}$ is the *i*th model output scalar value. The confusion matrix obtained after validating the model with a validation collection of 6407 images is used to measure the confusion matrix. The confusion matrix is used to evaluate the classification models' results. The training curve of the three pretrained models is shown in Figures 9–11. The graph is plotted for each epoch versus the training loss and accuracy. The graph is interpreting the training loss and training accuracy calculated versus the epoch. VGG16 model is trained for 30 epoch among the training dataset, and the model is proved to be converged after 15 epoch with accuracy ranges between 96%. After the 30 epochs, the model is provided with top_1 accuracy of 96.62%, top_5 accuracy of 100%, and validation loss of 0.18. The ResNet-18 model is proved to provide less training accuracy of 78.83% and high training loss of 0.58 after the epoch of 30. The GoogLeNet model has obtained a top_1 accuracy of 91.21%, top_5 accuracy of 100%, and training loss of 0.21.

After the model training is completed, the models are validated with the validation dataset, and the confusion matrix is drawn out of it. Figures 12–14 represent the confusion matrices of the three pretrained models validated on the validation dataset. The confusion matrix is drawn with truth data and classifier results. From the confusion matrix, the True Positive Value (TPV), False Positive Value (FPV), True Negative Value (TNV), and False Negative Value (FNV) are calculated. The diagonal elements represent the TPV of the corresponding class. The different performance metrics such as top_1 accuracy, top_5 accuracy, recall, precision, and Cohen's Kappa score are calculated using equations mentioned in Table 2.

The kappa coefficient is the de facto norm for assessing rater agreement, as it eliminates predicted agreement due to chance. Cohen's kappa value is obtained by equation (3), where *G* denotes overall correctly predicted classes, *H* denotes the total number of elements, *c*_*l*_ denotes the overall times class l that was predicted, and *s*_*l*_ denotes overall times class l occurred [33].

(3) $$\begin{array}{c} \text{CK}=\frac{G\times H-\sum_{l}^{L}c_{l}\times s_{l}\;}{H^{2}-\sum_{l}^{L}c_{l}\times s_{l}\;}. \end{array}$$

The kappa coefficient is used when the number of classes more to determine its classification performance. The value interprets the kappa score ranges from 0 to 1, and their interpretation is provided in Table 3.

All the pretrained models are trained from scratch to classify gastrointestinal tract diseases using the Kvasir v2 dataset, and results are reported in Table 4. The VGG16 methods outperformed all the other pretrained models in terms of all classification metrics. The model achieved the highest top_1 classification accuracy of 96.33% compared to the ResNet-18 and GoogLeNet models. The model also performs a perfect recall and precision with 96.37% and 96.5%, respectively. The GoogLeNet model achieved better accuracy over ResNet-18 with top_1 classification accuracy. The kappa coefficient is calculated for models, from that VGG16 and GoogLeNet model provided almost perfect agreement with the value of 0.96 and 0.89, respectively. Because of the high miss classification of diseases in the category dyed lifted polyps, dyed resection margins, esophagitis, standard *Z*-line, and polyps, ResNet-18 offers very low metrics in terms of all classification metrics. Owing to the injection of liquid underneath the polyp, the model is unable to correctly distinguish dyed lifted polyps and dyed resection margins, making the model more difficult to classify. The VGG16 and GoogLeNet models are proved to provide better accuracy in classifying the GIT diseases. However, the model is more difficult to identify because of the interclass similarity between dyed lifted polyps and dyed resection margins, as well as the intraclass similarity between standard *Z*-line and esophagitis.

The MCC is a more reliable statistical rate that produces a higher rate when the prediction results are good in all four values TPV, FPV, TNV, and FNV. It is calculated using equation (4).

(4) $$\begin{array}{c} \text{MCC}=\frac{G\times H-\sum_{l}^{L}c_{l}\times s_{l}\;}{\sqrt{\left(H^{2}-\sum_{l}^{L}c_{l}^{2}\right)\;\left(H^{2}-\sum_{l}^{L}s_{l}^{2}\right)}\;}. \end{array}$$

Using the Kvasir v2 datasets, the modified VGG16 model is compared with other models in classifying GIT diseases based on results reported in the article showed in Table 5. The Densenet-201 and ResNet-18 models that are reported in the reference [34] achieved an accuracy of 90.74% and 88.43%. Both the models are trained for more than 400 epochs, and it has taken roughly 10 hours to complete training. The model reported in [35] has provided an accuracy of 96.11%, which is very close to the proposed method reported in Table 5. But the said model uses the three stages model of baseline, Inception-V3, and VGG model, which requires high computation power and obtained the Matthews Correlation Coefficient (MCC) of 0.826. In [36], the CNN and transfer learning model is proposed classify GIT diseases using global features. The model achieves an accuracy of 93.7% with an MCC value of 0.71. The logistic model tree proposed in the reference uses the handcrafted features using 4000 images and achieves an accuracy of 94.2% but with poor MCC values of 0.72 [29]. The person's significant disadvantage should be knowledge of feature extraction and feature selection techniques. The modified pretrained model VGG16 obtained the MCC value of 0.95, which outperforms all the other models. From the MCC of all the states of the method, we found that the modified VGG16 method proves to be a perfect agreement for classifying GIT diseases.

The time complexity of the modified pretrained model is compared with the other models in classifying the GIT diseases. The proposed models VGG16, GoogLeNet, and ResNet-18 reported the training time of 1 hour 50 minutes, 1 hour, 7, and 57 minutes, respectively. The literature found that DenseNet-201 [34] and ResNet-18 [34] have been trained for more than 10 hours. The ROC curve in Figure 15(a) depicts the tradeoff between true-positive and false-positive rates. The ROC curve shows the performance of the classification model at different classification thresholds. It is plotted at different classification thresholds. The ROC is drawn for the eight classes to determine the better threshold for each category. The curve that fits the top left of the corner indicates the better performance of classification. Occlusion sensitivity is used to assess the deep neural network's sensitivity map to identify the image input area for predicted diagnosis. The heat map for test data is shown in Figure 15(b). This test procedure identified the region of interest, which was crucial in the development of the VGG16 model. The model's occlusion sensitivity map is visualized to determine the areas of greatest concern when evaluating a diagnosis. The occlusion test's greatest advantage is that it shows unresponsive insights into neural network decisions, also known as black boxes. The algorithm has been disfigured without disrupting its performance since the evaluation was performed at the end of the experiment.

## 6. Conclusion

These findings show that the most recent pretrained models, such as VGG-16, ResNet-18, and GoogLeNet, can be used in medical imaging domains such as image processing and analysis. CNN models can advance medical imaging technology by offering a higher degree of automation while also speeding up processes and increasing efficiency. The algorithm in this study obtained a state-of-the-art result in gastrointestinal tract disease classification, with 96.33% and equally high sensitivity and specificity. Transfer learning is helpful for various challenging tasks and is one solution to computer vision problems for which only small datasets are often accessible. Medical applications demonstrate that advanced CNN architectures can generalize and acquire very rich features, mapping information on images similar to those in the ImageNet database and correctly classifying very different cases. Compared to the various machine learning and deep learning models used to classify gastrointestinal tract disease, the VGG16 model achieves better results of 96.33% accuracy, 0.96 Cohen's kappa score, and 0.95 MCC. The requirement of manually marking data is the algorithm's weakest point. As a result, the network could inherit some flaws from an analyst, as diagnosing diseases correctly is difficult even for humans in many cases. Using a larger dataset labelled by a larger community of experts will be one way to overcome this limitation.

## Figures and Tables

**Figure 1:** Workflow for GIT disease classification from wireless endoscopy.

**Figure 2:** Sample images of Kvasir v2 dataset with eight different classes.

**Figure 3:** Dataset distribution among the different classes.

**Figure 4:** VGG16 architecture for gastrointestinal tract disease classification.

**Figure 5:** ResNet-18 architecture for gastrointestinal tract disease classification.

**Figure 6:** Inception module.

**Figure 7:** GoogLeNet architecture for gastrointestinal tract disease classification.

**Figure 8:** Augmented Kvasir v2 dataset.

**Figure 9:** VGG16 training graph for GIT classification.

**Figure 10:** ResNet-18 training graph for GIT classification.

**Figure 11:** GoogLeNet training graph for GIT classification.

**Figure 12:** VGG16 confusion matrix for GIT classification.

**Figure 13:** ResNet-18 confusion matrix for GIT classification.

**Figure 14:** GoogLeNet confusion matrix for GIT classification.

**Figure 15:** (a) VGG16 ROC for GIT classification. (b) Heat map for test data.

**Table 1:** Kvasir v2 dataset details.

Disease name	Class	Description
Dyed lifted polyps	Class 0	The raising of the polyps decreases the risk of damage to the GI wall's deeper layers due to electrocautery. It is essential to pinpoint the areas where polyps can be removed from the underlying tissue.
Dyed resection margins	Class 1	The resection margins are crucial for determining whether or not the polyp has been entirely removed.
Esophagitis	Class 2	Esophagitis is a condition in which the esophagus becomes inflamed or irritated. They appear as a break in the mucosa of the esophagus.
Normal-cecum	Class 3	In the lower abdominal cavity, the cecum is a long tube-like structure. It usually gets foods that have not been digested. The significance of identifying the cecum is that it serves as evidence of a thorough colonoscopy.
Normal-pylorus	Class 4	The pylorus binds the stomach to the duodenum, the first section of the small bowel. The pylorus must be located before the duodenum can be instrumented endoscopically, which is a complicated procedure.
Normal-*Z*-line	Class 5	The *Z*-line depicts the esophagogastric junction, which connects the esophagus's squamous mucosa to the stomach's columnar mucosa. It is vital to identify *Z*-line to determine whether or not a disease is available.
Polyps	Class 6	Polyps are clumps of lesions that grow within the intestine. Although the majority of polyps are harmless, a few of them can lead to colon cancer. As a result, detecting polyps is essential.
Ulcerative colitis	Class 7	The entire bowel will affect by ulcerative colitis (UC) affects which can lead to long-term inflammation or bowel wounds.

**Table 2:** Classification metrics.

Metric	Equation
Accuracy (ACC)	$\frac{\text{TPV}+\text{TNV}}{\text{TPV}+\text{TNV}+\text{FNV}+\text{FPV}}$
Precision	$\frac{\text{TPV}}{\text{TPV}+\text{FPV}}$
Recall	$\frac{\text{TPV}}{\text{TPV}+\text{FNV}}$
F1-measure	$2*\frac{\text{Precision}.\text{Recall}}{\text{Precision}+\text{Recall}}$

**Table 3:** Cohen's kappa interpretation.

Value ranges	Interpretation (agreement)
0	No
0.01 to 0.20	Minor
0.21 to 0.40	Moderate
0.41 to 0.60	Reasonable
0.61 to 0.80	Significant
0.81 to 1.00	Perfect

**Table 4:** Performance analysis of pretrained models on GIT classification.

Model name	Top_1 ACC (%)	Top_5 ACC (%)	Recall (%)	Precision (%)	F1-measure (%)	Kappa score
VGG16	96.33	100	96.37	96.50	96.50	0.96
GoogLeNet	90.27	100	90.33	90.27	90.37	0.89
ResNet-18	78.77	99.99	78.91	78.77	78.75	0.75

**Table 5:** Performance analysis of proposed method with existing models.

Method	Accuracy
DenseNet-201 [34]	90.74
ResNet-18 [34]	88.43
Baseline+Inceptionv3 + VGGNet [35]	96.11
Ensemble model [36]	93.7
Logistic regression tree [29]	94.2
Proposed method	96.33

## Data Availability

The data used to support the findings of this study are included within the article.
